# A 1 year course of starch- and sucrose-reduced diet used by irritable bowel syndrome patients with diarrhoea and the effect of genetic variants

**DOI:** 10.3389/fnut.2023.1268538

**Published:** 2023-10-26

**Authors:** Koldo Garcia-Etxebarria, Lucía Gayoso, Teresa Arzallus, Isabel Montalvo, Jacobo Lizasoain, Arantzazu Izagirre, Ander Ezkurra, Mauro D’Amato, Usune Etxeberria, Luis Bujanda

**Affiliations:** ^1^Biodonostia, Gastrointestinal Genetics Group, Donostia-San Sebastián, Spain; ^2^Centro de Investigación Biomédica en Red de Enfermedades Hepáticas y Digestivas (CIBERehd), Barcelona, Spain; ^3^Technology Center in Gastronomy, Basque Culinary Center, BCC Innovation, Donostia-San Sebastián, Spain; ^4^Basque Culinary Center, Faculty of Gastronomic Sciences, Mondragon Unibertsitatea, Donostia-San Sebastián, Spain; ^5^Biodonostia, Gastrointestinal Diseases Group, Universidad del País Vasco (UPV/EHU), Donostia-San Sebastián, Spain; ^6^Gastrointestinal Genetics Lab, CIC bioGUNE, Basque Research and Technology Alliance, Bilbao, Spain; ^7^Ikerbasque, Basque Foundation for Sciences, Bilbao, Spain; ^8^Department of Medicine and Surgery, LUM University, Bari, Italy

**Keywords:** diet, irritable bowel syndrome, long-term follow-up, intervention, genetics

## Abstract

**Background:**

Irritable bowel syndrome is a heterogeneous syndrome and it is difficult to find an effective treatment. Previously, a starch- and sucrose-reduced diet (SSRD) demonstrated promising short-term outcomes. It was proposed that genetic variants in the sucrose-isomaltase gene might influence this success. Our aim in this work was to extend the follow-up study to 1 year and to analyse the effect of the genetic variants of genes involved in starch and sucrose metabolism.

**Methods:**

IBS-SSS questionnaire, IBS-QoL questionnaire and questionnaires about adherence, difficulty and food assessment were sent to 34 patients after 6 months and 1 year after the end of the dietary intervention. In addition, 11 genes involved in sucrose and starch metabolism were sequenced.

**Results:**

Twenty-three participants responded to the 6 months follow-up and 16 to the 1 year follow-up. IBS-SSS total value increased 59.71% in the 6 months follow-up compared with the end of the intervention (*p* = 0.0018), and 55.39% in the 1 year follow-up (*p* = 0.0166); while IBS-QoL score decreased 24.09% (*p* = 0.0002) and 18.07% (*p* = 0.0022), respectively. The adherence decreased by 29.11% (*p* = 4.8 × 10^−5^) and 27.21% (*p* = 0.0054), respectively. In addition, carriers of pathogenic variants on the *SI* gene showed a slightly better performance than non-carriers. Finally, the participants showed less satisfaction over time with 18 allowed foods in the diet.

**Conclusion:**

Over time the SSRD is difficult to follow and the genotype might affect the performance of the diet. Since this diet could be a promising therapeutic option, a larger cohort needs to be analysed to validate the results and to compare it with other diets.

## 1. Introduction

Irritable bowel syndrome (IBS) is a condition that could be developed by between 5% and 20% of the general population, depending on the population and region analysed and diagnosis criteria used (1, 2). IBS is presented with symptoms in the lower gastrointestinal tract, such as abdominal pain and altered bowel habits (1, 2). Due to those symptoms and the difficulty of managing them, IBS could be a high burden for the patients and, therefore, for the health system, since IBS patients have greater use of the health system (1, 2). In addition, since the aetiology of IBS is unknown, it is defined as a heterogeneous syndrome and there is a lack of reliable biomarkers (1–3). Thus, it is difficult to find effective treatments for IBS.

Previously, a diet based on reducing the intake of sucrose and starch was used to treat the symptoms of IBS (4). We conducted a pilot study following that approach on patients of IBS suffering from diarrhoea and promising results were obtained (5): a high percentage of patients responded to the dietary intervention, there was an improvement in the symptoms (according to the Irritable bowel syndrome-symptom severity scale questionnaire) and the quality of life (according to the irritable bowel syndrome quality of life questionnaire), the adherence was high and the results were kept in the 2 months follow-up (5). In addition, the role of the sucrose-isomaltase (*SI*) gene in those patients was meta-analysed and the possible effect of hypomorphic variants of the *SI* gene in the success of the starch- and sucrose-reduced diet was suggested (6).

Nevertheless, it is important to assess the effect and adherence of a diet in the long term. For example, the long-term follow-ups of a low FODMAP diet used in IBS patients showed that the effect on the symptoms remains and the adherence is high (7–11). Thus, it should be assessed the long-term effect of the starch- and sucrose-reduced diet.

Considering the previous points, in this work, we have extended the follow-up of the patients who participated in the pilot study to 1 year; and we have analysed the effect of the *SI* gene and an additional 10 genes involved in sucrose and starch metabolism in the results of the follow-up period.

## 2. Materials and methods

### 2.1. Participants

This work is a follow-up of a dietary intervention that was carried out previously (5). Briefly, patients diagnosed with diarrhoea-predominant IBS in the Gastroenterology service of Hospital Universitario Donostia (Spain) were invited to participate in that intervention and the patients filling the inclusion criteria (age between 18 and 70, at least weekly abdominal pain related to bowel habit in the past 3 months, altered bowel habit and more than 175 points in the Spanish version of irritable bowel syndrome-symptom severity scale questionnaire) carried out a 4 weeks starch- and sucrose-reduced diet.

This study was approved by the Local Ethics Committee (Comité de Ética del Área Sanitaria de Gipuzkoa, code: BUJ-NUT-2019-01).

### 2.2. Questionnaires

Two months, six months and one year after the end of the intervention follow-up questionnaires were sent by post to the participants: the Spanish version of the irritable bowel syndrome-symptom severity scale (IBS-SSS) questionnaire (12), the Spanish version of irritable bowel syndrome quality of life (IBS-QoL) questionnaire (13), questions about dietary adherence (0 to 10 score), the difficulty to follow the dietary protocol (0 to 10 score), and the satisfaction with allowed foods (3: good, 2: regular; 1: bad).

### 2.3. Sequencing

Using Illumina Design Studio, we designed an AmpliSeq DNA assay for targeted next-generation sequencing (NGS) of all coding exons of the following 11 genes involved in sucrose and starch metabolism: *TAS1R3*, *SLC2A5*, *AMY2B*, *TAS1R2*, *TREH*, *LCT*, *SLC5A1*, *SI*, *SLC2A2*, *MGAM*, *MGAM2*. The amplicons were sequenced using 150 bp paired-end reads in an Illumina NextSeq machine.

The raw reads were processed following the GATK best practices (14). Briefly, raw reads were QCed using Trimmomatic (v 0.39) (15), mapped against hg38 human genome assembly using BWA (v 0.7.17) (16), marking the duplicates using Picard (v 2.27.1) (17), and recalibrating the qualities and calling the variants using GATK (v 4.2.6.1) (18). Then, only variants with a minimum sequence depth of 20 and quality of 20 were kept.

The kept variants were annotated using ANNOVAR (v. 2020-06-08) (19) and variants with CADD value >20 or M-Cap value >0.025 were annotated as pathogenic variants, following the cut-off suggested by the authors of those pathogenicity prediction algorithms (20).

### 2.4. Statistical analyses

For all the questionnaires, a *t*-test was used to compare each follow-up time point with the values at the end of the intervention and previous to the dietary intervention; or with the values at the end of the intervention in the case of adherence, difficulty and satisfaction. The effect size of the *t*-test was calculated using Cohen’s *d* using the package rstatix^1^ of R language (21).

In addition, the improvement of IBS-SSS value (the difference between the value previous to the dietary intervention and the value of each follow-up time point) and adherence was compared stratified by carriership of pathogenic variants only in *SI* gene, in *SI* + other gene, only in another gene against non-carriers of pathogenic variants using a Mann–Whitney *U* test. The effect size was calculated using Cliff’s Delta estimate using the package “effsize” (22) of R language.

The R language and its ggplot2 package (23) were used to carry out the statistical analyses and graphics.

All methods were performed following relevant guidelines and regulations including the Declaration of Helsinki.

## 3. Results

Previously, 34 IBS patients with diarrhoea participated in a dietary intervention based on a starch- and sucrose-reduced diet and the 2 months follow-up was completed by 22 patients (5). In this study, we have extended the follow-up time points to 6 months and 1 year. The former was completed by 23 participants (67.65% of the IBS patients who completed the dietary intervention) and the latter by 16 participants (47.06%) (Figure 1A and Table 1).

**Figure 1:** Results of follow-up questionnaires. **(A)** Number of participants that responded in each time-point. **(B)** Total IBS-SSS score values. Black dots, individual results; in blue, the mean value; in shadowed blue, 95% of the confidence interval. *p*, the *p*-value of the *t*-test; Cohen’s *d*, effect size of *t*-test and 95% of the confidence interval, <0.2 negligible effect, 0.2–0.5 small effect, 0.5–0.8 moderate effect, >0.8 large effect. **(C)** Results of each IBS-SSS question. **(D)** Total IBS-QoL score values. Black dots, individual results; in blue, the mean; in shadowed blue, 95% of the confidence interval. *p*, the *p*-value of the *t*-test; Cohen’s *d*, effect size of *t*-test and 95% of the confidence interval, <0.2 negligible effect, 0.2–0.5 small effect, 0.5–0.8 moderate effect, >0.8 large effect. **(E)** Results of each IBS-QoL domain. Adherence and difficulty of the diet. **(F)** Adherence to the diet. Black dots, individual results; blue lines, median value. *p*, the *p*-value of the *t*-test; Cohen’s *d*, effect size of *t*-test and 95% of the confidence interval, <0.2 negligible effect, 0.2–0.5 small effect, 0.5–0.8 moderate effect, >0.8 large effect. **(G)** Difficulty complying with the diet. Black dots, individual results; blue lines, median value. *p*, the *p*-value of the *t*-test; Cohen’s *d*, effect size of *t*-test and 95% of the confidence interval, <0.2 negligible effect, 0.2–0.5 small effect, 0.5–0.8 moderate effect, >0.8 large effect.

**Table 1:** Demographics of the participants.

	End of the intervention	2 months follow-up	6 months follow-up	1 year follow-up
*N*	34	22	23	16
Female:Male	21:13 (62.76%:37.24%)	14:8 (63.64%:36.36%)	16:7 (69.56%:30.43%)	11:5 (68.75%:31.25%)
Age (SD)	42.83 (13.94)	42.77 (13.62)	43.52 (13.02)	44.87 (14.2)
Current smokers	13 (38.23%)	6 (27.27%)	7 (30.43%)	4 (25%)
Allergies	3 (8.82%)	2 (13.64%)	2 (8.69%)	2 (12.5%)
Intolerances	4 (11.76%)	1 (4.55%)	3 (13.04%)	1 (6.25%)

The completion of the follow-up questionnaires was irregular and some patients that did not complete the questionnaires in one follow-up time point completed them in the next. Thus, 14 patients completed the follow-up questionnaires in the three time points, 5 in the 2 months follow-up and 6 months follow-up, 2 in the 6 months follow-up and 1 year follow-up, 2 in the 2 months follow-up only and 2 the 6 months follow-up only.

Moreover, the demographics of the participants showed slight differences between different time points. Those differences were especially clear in the female:male ratio, where more female participants answered the questions; and the proportion of current smokers, which decreased over time.

### 3.1. Symptoms, quality of life and diet evaluation

The more time passed from the end of the intervention, the total value of IBS-SSS increased compared to the end of the intervention, although it did not equal the value before the start of the intervention (Figure 1B). The total value of IBS-SSS in the 6 months follow-up (mean value of 222 ± 92) and 1 year follow-up (mean value of 216 ± 101) was significantly higher compared to the end of the intervention (mean value of 139 ± 95; *p* = 0.0018 and *p* = 0.0166, respectively), that is, an increase of total IBS-SSS value of 59.71% and 55.39%, respectively. Compared with before the dietary intervention, the values were significantly lower (mean value of 291 ± 70; *p* = 0.0041 and *p* = 0.0136, respectively). In both cases, the effect of the *t*-test was moderate to large. It has to be pointed out that this change in the IBS-SSS questionnaire was similar to all the questions (Figure 1C and Supplementary Table S1).

In the case of total IBS-QoL Score, the value was significantly lower in the 6 months follow-up (mean value of 63 ± 20, *p* = 0.0002) and 1 year follow-up (mean value of 68 ± 16, *p* = 0.0022) compared to the end of the intervention (mean value of 83 ± 14) and the effect was large (Figure 1D). This decrease represents 24.09% and 18.07% of the total IBS-QoL score compared to the end of the intervention, respectively. Compared with the values before the intervention (mean value of 57 ± 19), although the mean values in the 6 months follow-up and 1 year follow-up were higher (an increase of 10.53% and 19.29% respectively), the difference was not significant (Figure 1D). These worst values of IBS-QoL were observed in all the domains that this questionnaire analyses (Figure 1E and Supplementary Table S2).

Finally, the adherence in the 6 months follow-up (mean value of 5.6 ± 2) and 1 year follow-up (mean value of 5.75 ± 2.5) was significantly lower (*p* = 4.8 × 10^−5^ and *p* = 0.0054, respectively) than the end of the intervention (mean value of 7.9 ± 1.4), and the effect was large (Figure 1F). That is, the adherence at the 6 months follow-up decreased 29.11% and 27.21% at 1 year follow-up compared with the end of the diet. In the case of the difficulty, there was not any significant change: 5.8 (±2.7) at the end of the intervention, 6.2 (±2.1) at the 6 months follow-up, and 5.8 (±2.6) at the 1 year follow-up (Figure 1G).

### 3.2. Effect of the genotype

We classified the participants according to the carriership of pathogenic variants in the *SI* gene, and another 10 genes involved in sucrose and starch metabolism. Then, we observed how they responded to the intervention at the different follow-up time points.

At the end of the intervention and in the three time points of the follow-up (2 months, 6 months and 1 year), the participants carrying pathogenic variants on the *SI* gene showed a better improvement (the difference of the IBS-SSS value between the start of the intervention and a given time point) in the total IBS-SSS score (Figure 2A and Supplementary Table S3): a mean value of 147.5 (±145) at 2 months follow-up, 117 (±93) at 6 months follow-up and 212 (±61) at 1 year follow-up. In the case of participants with pathogenic variants in *SI* and additional genes or in genes rather than *SI*, the improvement was lower than in the carriers of pathogenic variants only in *SI* (Figure 2A and Supplementary Table S3). In addition, the few participants without pathogenic variants showed worse values in the follow-up time points (Figure 2A): a mean value of −9 (±104) at 2 months follow-up, −49 (±92) at 6 months follow-up and −54 (±21) at 1 year follow-up.

**Figure 2:** Results stratified by carriership of pathogenic variants of genes involved in sucrose and starch metabolism. **(A)** IBS-SSS score improvement, the difference between a time point and before the start of the intervention. **(B)** Adherence.

In the case of adherence to the dietary protocol, a similar trend was observed (Figure 2B and Supplementary Table S4): the adherence of carriers of pathogenic variants on *SI* was 7 (±2.16) at 2 months follow-up, 7.4 (±1.14) at 6 months follow-up and 7.2 (±1.9) at 1 year follow-up, while the adherence of the participants without pathogenic variants was 5 (±4.36) at 2 months follow-up, 4.3 (±3.79) at 6 months follow-up and 3 (±4.24) at 1 year follow-up. In addition, the values of pathogenic variants in *SI* and additional genes or in genes rather than *SI* were intermediate (Figure 2B and Supplementary Table S4).

Although the majority of these differences between the groups was not significant (Supplementary Tables S3, S4), the difference in the improvement of IBS-SSS between carriers of pathogenic variants in any gene and the non-carriers was significant at 1 year follow-up (*p* = 0.0385) and the effect was large (Cliff’s Delta = −0.82, 95% of confidence interval =−0.98–0.11).

### 3.3. Food evaluation

The participants were asked to evaluate how much they liked the 86 foods that were allowed to eat in the dietary protocol. Overall, the participants liked those foods but the satisfaction of 18 foods significantly decreased at one or more time points (Figure 3 and Supplementary Table S5).

**Figure 3:** Satisfaction of the participants with allowed food (3: good, 2: regular; 1: bad). Bar plots depict the mean value at each time point; the lines depict the standard deviation; *p*, the *p*-value of the *t*-test. Only significant results (*p* < 0.05) are shown.

Four foods showed a lower satisfaction in 2 months, 6 months and 1 year time points than at the end of the intervention: kiwi (from 3 to 2.56 ± 0.73, 2.53 ± 0.74 and 2.25 ± 0.75, respectively), brussels sprout (from 3 to 2.29 ± 0.76, 2.14 ± 0.69 and 1.86 ± 0.38, respectively), cucumber (from 3 to 2.56 ± 0.53, 2.4 ± 0.7 and 2.38 ± 0.52, respectively) and milk (from 2.97 ± 0.18 to 2.5 ± 0.89, 2.29 ± 0.92 and 2.43 ± 0.76, respectively). In addition, artichoke, collard greens, mushrooms and pepper in 6 months and 1 year time points; and pear, broccoli, cabbage, spinach, lettuce, tomato, butter and lamb in one time point (Figure 3 and Supplementary Table S4).

## 4. Discussion

Previously we reported the promising results of a pilot study that analysed the effect of starch- and sucrose-reduced diet (SSRD) and a follow-up of 2 months in patients of IBS with diarrhoea (5). In addition, it was suggested that the *SI* gene could affect those results since carriers of hypomorphic variants of the *SI* gene can benefit more from the SSRD (6). Now, we have extended the follow-up time to 1 year and the analysis of the genotype to an additional 10 genes involved in sucrose and starch metabolism.

First of all, the more time passed since the end of the intervention, the fewer people sent the follow-up questionnaires, getting the response of less than half of the participants at 1 year follow-up. For example, in a follow-up study of the application of a low FODMAP diet in IBS and inflammatory bowel disease with coexisting IBS patients, questionnaires were sent by mail to 348 patients and 180 (52%) answered one or more questionnaires (7). In addition, in other follow-up studies of the use of a low FODMAP diet in IBS patients, the rates were 103 responses from 375 eligible participants (27%) (8), 224 from 499 (45%) (11), 90 from 234 (38%) (10), and 41 from 73 (56%) (9). In this sense, the drop in the response rate in our work seems to be in line with the results obtained in other follow-up studies. As a consequence, we could conclude that only the participants who responded better to the diet could send their questionnaires. However, the answers obtained from the participants were heterogeneous (from participants whose values remain similar to the end of the intervention to participants whose values worsen) and that makes us confident that we have avoided selection or survival biases. Anyway, the drop in the responses is a limitation and raises the question if they have not sent the follow-up questionnaires because they think that the diet is not suitable for them or due to other external reasons, as it was a concern in other follow-up studies from dietary interventions in IBS (7, 8, 11).

We are aware that as a consequence of the drop in the responses, our sample size is limited and, therefore, the conclusions that we can make from the results are also limited. However, although the statistical power was limited, we were able to detect significant differences between the follow-up time points and the start and end points of the intervention. Thus, we could state that, over time, the symptoms deteriorate and that the quality of life also worsens, although these results are still better than the values obtained before the beginning of the intervention. When a low FODMAP diet has been used in IBS patients, in the long-term the improvement of the symptoms was not as high as at the end of the intervention, although the symptoms did not deteriorate as significantly as in our study (7–11). In this sense, the impediment seems to be the adherence since it was lower at 1 year follow-up compared to the end of the intervention and the difficulty of following the diet did not change. In the low FODMAP diet, the reintroduction and personalization phases help to maintain adherence to the diet (7–11). Thus, it might be possible to maintain adherence to the SSRD by designing complementary strategies to facilitate adherence over time.

Another factor that could explain the results obtained is the carriership of pathogenic variants of genes involved in sucrose and starch metabolisms. Previously, several works have analysed the role of *SI* in IBS, especially with diarrhoea (24–26), and its effect on dietary interventions (6, 27). Unfortunately, our limited sample size did not allow us to have clear evidence, although it seems to be a trend where the carriers of pathogenic genetic variants of the *SI* gene show better performance than the non-carriers. The majority of the participants were carriers of a pathogenic variant in genes involved in starch and sucrose metabolisms and that could partially explain the effectiveness of the diet at the end of the intervention in our cohort, although it is not enough to keep the efficacy over time. Furthermore, the participants with pathogenic genetic variants only in the *SI* gene showed slightly better performance than those carrying pathogenic genetic variants in other genes or combined with *SI*. It could be possible that the symptoms of patients could be triggered by other foods in those participants (for example, carriers of pathogenic variants in lactase could have lower results since milk is not restricted in SSRD).

Moreover, we asked the participants about their satisfaction with the foods they were allowed to eat, to know if there were foods that they disliked over time. Since one of the main reasons for not following a low FODMAP diet in IBS over time was the bland taste (7), it was important to detect if the liking of the allowed foods was steady. In one or more time points 18 foods showed less satisfaction than at the end of the intervention and that may suggest that the participants could avoid the consumption of those foods, making it more difficult to adhere to the diet. One of the foods with lower punctuation in satisfaction was milk and that could be in line with the lower effectiveness of the diet observed in patients who were carriers of pathogenic variants in other genes than *SI*. Thus, it seems that the role of those foods in the SSRD should be adjusted to facilitate adherence to the diet.

On the whole, we concluded that it is difficult to follow the SSRD in the long term, which affects the improvements in the symptoms and quality of life, although the results obtained are better than the ones obtained before the beginning of the dietary intervention. We have observed that the carriership of pathogenic genetic variants in genes involved in starch and sucrose metabolism might have an effect on the performance of the diet over time, but we were not able to have clear evidence, since the results were not significant. However, we still think that SSRD could be a promising therapeutic option for IBS patients with diarrhoea and it is worth applying this strategy in a larger cohort, to have enough statistical power to compare it with other dietary interventions and to elucidate the role of genetic variants in the response to the diet.

## Data availability statement

The datasets presented in this article are not readily available because sequencing data cannot be make available due to ethical limitations. Requests to access the datasets should be directed to KG-E, koldo.garciaetxebarria@biodonostia.org.

## Ethics statement

The studies involving humans were approved by Comité de Ética del Área Sanitaria de Gipuzkoa. The studies were conducted in accordance with the local legislation and institutional requirements. The participants provided their written informed consent to participate in this study.

## Author contributions

KG-E: Conceptualization, Data curation, Formal analysis, Investigation, Methodology, Visualization, Writing – original draft, Writing – review & editing. LG: Conceptualization, Methodology, Resources, Writing – review & editing. TA: Resources, Writing – review & editing. IM: Resources, Writing – review & editing. JL: Resources, Writing – review & editing. AI: Resources, Writing – review & editing. AE: Resources, Writing – review & editing. MD’A: Conceptualization, Funding acquisition, Methodology, Resources, Writing – review & editing. UE: Conceptualization, Methodology, Resources, Writing – review & editing. LB: Conceptualization, Funding acquisition, Investigation, Resources, Supervision, Writing – review & editing.

## Footnotes

^1^ https://CRAN.R-project.org/package=rstatix
